The article "Attrition of TCR Vα7.2+ CD161++ MAIT Cells in HIV-Tuberculosis Co-Infection Is Associated with Elevated Levels of PD-1 Expression" was published in 2015. Journal: PLoS One.

# Attrition of TCR Vα7.2+ CD161++ MAIT Cells in HIV-Tuberculosis Co-Infection Is Associated with Elevated Levels of PD-1 Expression

**DOI:** 10.1371/journal.pone.0124659

**Published:** 2015-04-20

**Authors:** Alireza Saeidi, Vicky L. Tien Tien, Rami Al-Batran, Haider A. Al-Darraji, Hong Y. Tan, Yean K. Yong, Sasheela Ponnampalavanar, Muttiah Barathan, Devi V. Rukumani, Abdul W. Ansari, Vijayakumar Velu, Adeeba Kamarulzaman, Marie Larsson, Esaki M. Shankar

**Affiliations:** 1 Tropical Infectious Diseases Research and Education Center (TIDREC), Department of Medical Microbiology, Faculty of Medicine, University of Malaya, Lembah Pantai, 50603 Kuala Lumpur, Malaysia; 2 Center of Excellence for Research in AIDS (CERiA), University of Malaya, Lembah Pantai, 50603 Kuala Lumpur, Malaysia; 3 Department of Biomedical Science, Faculty of Medicine, University of Malaya, Lembah Pantai, 50603 Kuala Lumpur, Malaysia; 4 Department of Molecular Medicine, Faculty of Medicine, University of Malaya, Lembah Pantai, 50603 Kuala Lumpur, Malaysia; 5 Department of Microbiology and Immunology, Emory Vaccine Center, 954 Gatewood Road, Atlanta, GA 30329, United States of America; 6 Molekylär Virologi, Institutionen för Klinisk Och Experimentell Medicin, Linköpings Universitet, 581 85 Linköping, Sweden; Karolinska Institutet, SWEDEN

## Abstract

Mucosal-associated invariant T (MAIT) cells are evolutionarily conserved antimicrobial MR1-restricted CD8^+^ T cells co-expressing the semi-invariant TCR Vα7.2, and are numerous in the blood and mucosal tissues of humans. MAIT cells appear to undergo exhaustion in chronic viral infections. However, their role in human immunodeficiency virus type 1 (HIV-1) mono-infection and HIV/tuberculosis (TB) co-infection have seldom been elaborately investigated. We conducted a cross-sectional study to investigate the frequencies and phenotypes of CD161^++^CD8^+^ T cells among anti-retroviral therapy (ART)/anti-TB therapy (ATT) treatment-naïve HIV/TB co-infected, ART/TB treated HIV/TB co-infected, ART naïve HIV-infected, ART-treated HIV-infected patients, and HIV negative healthy controls (HCs) by flow cytometry. Our data revealed that the frequency of MAIT cells was severely depleted in HIV mono- and HIV/TB co-infections. Further, PD-1 expression on MAIT cells was significantly increased in HIV mono- and HIV-TB co-infected patients. The frequency of MAIT cells did not show any significant increase despite the initiation of ART and/or ATT. Majority of the MAIT cells in HCs showed a significant increase in CCR6 expression as compared to HIV/TB co-infections. No marked difference was seen with expressions of chemokine co-receptor CCR5 and CD103 among the study groups. Decrease of CCR6 expression appears to explain why HIV-infected patients display weakened mucosal immune responses.

The article "Attrition of TCR Vα7.2+ CD161++ MAIT Cells in HIV-Tuberculosis Co-Infection Is Associated with Elevated Levels of PD-1 Expression" was published in 2015. Journal: PLoS One.

## Introduction

Human immunodeficiency virus type 1 (HIV-1) infection leads to dramatic loss of CD4^+^ T cells and increased systemic T-cell activation contributing to increased susceptibility to opportunistic infections (OIs), especially with *Mycobacterium tuberculosis* (MTB) [1–3]. MTB and HIV infections interfere and have a remarkable impact on each other’s pathogenesis [4]. Of note, HIV infection is the utmost risk factor for acquisition of MTB infection [5]. Clinical evidence suggests that despite long-term highly-active antiretroviral treatment (HAART), susceptibility to MTB infection is not fully repaired, and that loss of the CD4^+^ T cells is not the sole responsible mechanism [5, 6].

Mucosal-associated invariant T (MAIT) cells represent a distinct T-cell subset that accounts for ~1/3^rd^ of the CD8^+^ T-cell pool in the blood of healthy individuals [7–9]. MAIT cells express a semi-invariant Vα7.2-Jα33/12/20 T-cell receptor (TCR) that recognize antigens presented on the MHC class I-related (MR1) molecule [7, 9, 10]. CD161 is a C-type lectin-like receptor found on CD4^+^, CD8^+^, γδ T cells, and NK cells [11–14] and also within CD8^-^CD4^-^ T cells. The expression of CD161 helps distinguish three distinct subsets, viz., CD161^-^, CD161^+^, and CD161^++^ subsets [15, 16]. The CD161^++^CD8^+^ T cells reportedly produce IL-17A and IL-22, factors important in the maintenance of mucosal integrity and antibacterial immune responses [9, 16–18]. More recently, an important overlap between expression of CD161 and MAIT cells has been reported with ~80–90% of CD161^++^ cells co-expressing the canonical Vα7.2 TCR [11, 19]. MAIT cells express a range of chemokine receptors, which serves to explain its preferential localization and trafficking to the gut, but more prominently to the lungs and liver [9, 11, 20]. MAIT cells can be activated by MR1-ligand-TCR ligation or via exposure to IL-12 and IL-18 leading to release of pro-inflammatory cytokines and granzymes [10, 21–23]. MAIT cells also appear to have a role in host immune responses against MTB [15, 24].

MTB-infected individuals reportedly have lower frequencies of MAIT cells as compared with healthy individuals, although there appears to be limited difference in the frequencies between active and latent MTB infections [25]. MAIT cells from healthy individuals express significantly lower levels of activation markers (CD38, HLA-DR), inhibitory (TIM-3), and senescence markers (CD57) than those from HIV-infected individuals. Interestingly, evidence suggests that long-term anti-retroviral treatment (ART) has been shown to decrease HLA-DR and TIM-3 although this seldom seems to alleviate the expressions of CD38 and CD57 on MAIT cells [26]. Here, we investigated how the CD161^++^CD8^+^ T-cell populations were affected HIV infection and by HIV/MTB co-infection, especially in the context of ART/ATT therapy. We also sought to understand the molecular basis behind potential MAIT cell exhaustion, and investigate the frequency of expression of programmed cell death protein 1 (PD-1), which has a concrete role in the exhaustion of classical CD8^+^ and CD4^+^ T cells in HIV disease.

The article "Attrition of TCR Vα7.2+ CD161++ MAIT Cells in HIV-Tuberculosis Co-Infection Is Associated with Elevated Levels of PD-1 Expression" was published in 2015. Journal: PLoS One.

## Materials and Methods

### Ethics Statement

The protocols involving human subjects were approved by the Medical Ethics Committee (MEC) of University of Malaya Medical Centre (UMMC), Kuala Lumpur, Malaysia (MEC201311-0496), and conducted as per the guidelines of the International Conference on Harmonization Guidelines and Declaration of Helsinki. All participants provided written informed consent. The written consent form was approved by the ethics committee and signed by the subject or the subject's legally authorized representative. A copy of the document was given to the person signing the form. The entire consent process was approved by the MEC for conduct of the research.

### Patients

A total of 50 individuals with different infection statuses with HIV mono-infection or HIV/TB co-infection were recruited for a cross-sectional investigation in Kuala Lumpur, Malaysia. Healthy control (HC) individuals (HIV and TB negative) (n = 10), ART/TB treatment naïve HIV/TB co-infected patients (CPTN, n = 10), ART/ATT-treated HIV/TB co-infected patients (CPTP, n = 10), ART naïve HIV-infected patients (HVTN, n = 10) and HIV infected patients on ART (HVTP, n = 10). All individuals in the untreated infection groups were ART and TB therapy naïve, and all the treated patients had received treatment for two years. Co-infected patients were pulmonary TB cases identified by a positive sputum acid-fast bacilli (AFB) staining (Ziehl-Neelsen or auramine phenol staining) or sputum culture. All individuals defined as negative for TB were asymptomatic, commercial RD1-based ELISPOT-IFN-gamma (IFN-γ) assay negative and sputum smear and culture negative for MTB on induced sputum. HIV and MTB mono- and co-infected individuals were recruited at the Infectious Diseases Clinic of the University of Malaya Medical Centre (UMMC), Malaysia. HCs were defined as persons free from any viral infections (HBV, HCV and HIV), and TB infection. HC individuals were recruited at the Blood Transfusion Clinic of the UMMC. Descriptive and clinical data obtained from the participating subjects is shown in Table 1.

The article "Attrition of TCR Vα7.2+ CD161++ MAIT Cells in HIV-Tuberculosis Co-Infection Is Associated with Elevated Levels of PD-1 Expression" was published in 2015. Journal: PLoS One.

**Table 1:** Demographic, clinical and laboratory characteristics of study participants.

Study Groups	CPTN (n = 10)	CPTP (n = 10)	HVTN (n = 10)	HVTP (n = 10)	*p value*
Age, Mean (±SD), Years	41.9 (±7.2)	43.2 (±6.26)	37.3 (±7.95)	39.4 (±9.76)	0.3023^B^
Gender, N (%)					
Male	6 (60%)	8 (80%)	10 (100%)	9 (90%)	NA
Female	4 (40%)	2 (20%)	0 (0%)	1 (10%)	NA
**HIV Characteristics**					
Viral Load, copies/mlLog_10_ (Mean±SD)	5.118 (±0.4)	1.018 (±1.3)	5.096 (±0.5)	0.939 (±0.62)	<0.0001*** ^B^
**CD4** ^**+**^ **T-cell count, cells/mm** ^**3**^ **(Mean±SD)**	78.1 (±157.2)	264.56 (±174.6)	211 (±92.8)	430.8 (±194.6)	0.0004*** ^B^
<200 cells/mm^3^	26.89 (±35.4)	122.67 (±28.2)	117.25 (±61.9)	176.5 (±1.5)	0.0167* ^B^
>200 cells/mm^3^	539	335.5 (±173.8)	273.5 (±45.1)	494.375 (±164.7)	0.0427* ^B^
CD4^+^ T-cell count, N (%)					
<200 cells/mm^3^	9 (90%)	3 (33.3%)			0.0198^A^
>200 cells/mm^3^	1 (10%)	6 (66.7%)			
<200 cells/mm^3^			4 (40%)	2 (20%)	0.6285^A^
>200 cells/mm^3^			6 (60%)	8 (80%)	
**CD8** ^**+**^ **T-cell count, cells/mm** ^**3**^ **(Mean±SD)**	775.78 (±604.2)	939.22 (±625.4)	1107.3 (±421.4)	1113.5 (±408.8)	0.3642^B^
<800 cells/mm^3^	303.6 (±179.5)	513.6 (±255.061)	653 (±83.6)	769.67 (±23)	0.0369* ^B^
>800 cells/mm^3^	1366 (±392.5)	1471.25 (±537.95)	1410.1 (±248.9)	1260.8 (±407.6)	0.6804^B^
CD8^+^ T-cell count, N (%)					
<800 cells/mm^3^	5 (55.56%)	5 (55.56%)			1.000^A^
>800 cells/mm^3^	4 (44.44%)	4 (44.44%)			
<800 cells/mm^3^			4 (40%)	3 (30%)	1.000^A^
>800 cells/mm^3^			6 (60%)	7 (70%)	
**CD4** ^**+**^ **/CD8** ^**+**^ **T-cell ratio(Mean±SD)**	0.083 (±0.09)	0.412 (±0.3)	0.222 (±0.1)	0.4645 (±0.2)	0.002** ^B^
**TB Characteristics**					
Type of TB, N (%)					
Pulmonary	9 (90%)	7 (70%)			NA
Extra-Pulmonary	0 (0%)	2 (20%)			NA
Disseminated	1 (10%)	1 (10%)			NA

Footnotes: Statistical analyses performed using (A) Fisher’s Exact test and (B) Kruskal-Wallis non-parametric ANOVA test:

*p<0.05

**p<0.01

***p<0.001

CPTN: HIV/TB co-infection treatment naïve; CPTP: HIV/TB co-infection treatment positive; HVTN: HIV mono-infection treatment naïve; HVTP: HIV mono-infection treatment positive; NA: non- applicable. All values are expressed as mean ±SD.

### Peripheral Blood Mononuclear Cells

Ten milliliters (mL) of whole blood was collected from all subjects by venipuncture in lithium heparin BD Vacutainer (BD Biosciences, Franklin Lakes, USA). Within 3 hours of venipuncture, PBMCs were extracted from the whole blood samples by density-gradient centrifugation with FicollPaque Plus (Sigma-Aldrich) reagent. Cell viability was determined by 0.4% trypan blue vital staining procedure. PBMCs (1.5 x 10^6^ cells/mL) were immunostained immediately for MAIT cell markers following separation.

The article "Attrition of TCR Vα7.2+ CD161++ MAIT Cells in HIV-Tuberculosis Co-Infection Is Associated with Elevated Levels of PD-1 Expression" was published in 2015. Journal: PLoS One.

### MAIT Cell Immunophenotyping

All antibodies were pre-titrated to determine appropriate working concentrations. Immunostaining with periridin-chlorophyll protein (PerCp)-Cy5.5-conjugated anti-CD3 (BD Biosciences, clone UCHT1), allophycocynanin (APC)-H7-conjugated anti-CD8 (BD Biosciences, clone SK1) and APC-conjugated anti-CD161 (BD Biosciences, clone DX12) in the phenotypic characterization of MAIT cell was performed according to the protocol set by the commercial manufacturer (BD Biosciences). Surface staining for specific receptors was performed using monoclonal antibodies (mAbs) directed against: FITC-conjugated PD-1 (clone MIH4), phycoerythrin (PE)-conjugated CCR6 (clone 11A9), PerCp-Cy5.5-conjugated CCR5 (clone 3A9) and PE-conjugated TCR Vα7.2 (clone 3C10) (all mAbs procured from BD Biosciences). Immunostained samples were washed twice prior to acquisition on a FACS Canto II Immunocytometry system (BD Biosciences) and analyzed using FACS Diva software. Data were analyzed using FlowJo (version 9.3.1 and version 10). Doublets were excluded based on FSC-H and FSC-A, lymphocytes were identified based on FSC and SSC, and dead cells were excluded based on BD Horizon Fixable Viability Stain 510 (BD Biosciences). CD3^+^ and CD8^+^ T lymphocytes were identified. Fluorescence minus one (FMO) controls was used for optimal gating.

### Statistical Analysis

Mean and standard error of the mean (SEM) were used to describe each variables analyzed. Due to the sample size and the assumption that the sample population does not follow normal distribution, non-parametric unpaired t test (or Mann-Whitney U test) was selected for comparisons between the two independent groups. Two-sided Mann-Whitney tests for non-parametric data were used to compare the two groups. Differences were considered significant with *P<0.01, **P<0.001 and ***P<0.0001. Correlation analysis between CD161^++^CD8^+^ T-cell frequencies and HIV plasma viral load (PVL) was performed using the Spearman's rank correlation coefficient. All analyses were performed using the PRISM 5 software for Windows version 6.01(GraphPad, La Jolla, CA, USA).

## Results

### HIV Mono- and HIV/MTB Co-Infections Lead to Significant Depletion of CD161^++^CD8^+^ T Cells

The demographic, clinical and laboratory characteristics of the patient study groups are shown in Table 1. We first compared the frequency of CD161^++^CD8^+^ T-cell populations in the peripheral blood of four groups of patients with HIV mono-infection (ART and ART naïve groups), and HIV/TB co-infection (ART/ATT-treated and ART/ATT naïve groups) with HCs. For the sake of simplicity, here we have defined CD161^++^CD8^+^ T cells as CD161^++^/MAIT cells although a minority of the cells reportedly fall within the CD4^+^ and CD4^-^CD8^-^ (DN) subsets [7, 12]. CD161^++^/MAIT population was gated based on CD3^+^CD8^+^CD161^++^ cells (Fig 1A) whereas the differential expression of the TCR Vα7.2 was gated on the CD8^+^ T cell population by CD161^++^, CD161^+^ and CD161^-^ CD8^+^ T-cell subsets (Fig 1B). Our investigations of the PD-1 expression on CD161^+^CD8^+^ and CD161^++^CD8^+^ T cells derived from HCs, revealed that the expression was significantly increased (*P*<0.0001) on CD161^+^CD8^+^ T cells as compared to CD161^++^CD8^+^ T cells in HCs (Fig 1C). CCR6 expression was also significantly increased (*P*<0.0001) on CD161^++^CD8^+^ T cells compared to both CD161^-^CD8^+^ T cells and CD161^+^CD8^+^ T cells in HCs (Fig 1D).

The article "Attrition of TCR Vα7.2+ CD161++ MAIT Cells in HIV-Tuberculosis Co-Infection Is Associated with Elevated Levels of PD-1 Expression" was published in 2015. Journal: PLoS One.

**Fig 1:** Phenotypic properties of CD161^++^CD8^+^ T-cells. **(A)** Depiction of the gating strategy used: During acquisition, lymphocytes were selected on the basis of forward-scatter and side-scatter characteristics. MAIT cell subsets were gated from CD3, CD8 and CD161^bright^ cells, viz., CD3^+^CD8^+^CD161^++^ defined as MAIT cells. (**B)** Histograms (gated on the CD8^+^ T-cell population) show differential expression of TCR Vα7.2 by CD161^++^, CD161^+^ and CD161^-^CD8^+^ T cells from a representative sample from healthy controls (HC). **(C)** Collective data from 10 HCs demonstrated differential expression of PD-1 by CD161^++^, CD161^+^ and CD161^-^CD8+ T cells. **(D)** Aggregate data from 10 HCs demonstrated differential expression of CCR6 by CD161^++^, CD161^+^ and CD161^-^ CD8^+^ T-cell subsets. All graphs show median (red bars) and range (blue whiskers); *P* values are reported for two-sided Mann-Whitney tests with threshold for significance *P* = 0.02 after Bonferroni correction for 2 comparisons.

We also examined the frequencies of MAIT cells in the study population. Our results showed that HIV mono-infected ART naïve patients (median, 0.82%; range, 0.15–6.8; *P* = 0.05), HIV/TB co-infected patients treatment naïve (median, 0.75%; range, 0.08–2.3; *P* = 0.001), and HIV mono-infected patients with treatment (median, 1.38%; range, 0.16–3.4; *P* = 0.05) had a significantly lower number of MAIT cells as compared to HCs (median, 3.77%; range, 0.32–8.0) (Fig 2B). We also observed that a minority of the HCs had low number of MAIT cells while a minority of HIV-infected or HIV/TB co-infected patients had normal or nearly normal frequency of MAIT cells (data not shown). No significant changes were noted in frequencies of non-MAIT CD161^+^ (dim) CD8^+^ T-cells among the different groups (Fig 2C). The frequency of CD161^++^CD8^+^ T cells did not correlate with either PVL or CD4^+^ T-cell counts (r = 0.25; *P* = 0.1) (Fig 2D and 2E). We also observed in the healthy controls that the percentage of CD161^++^ T cells was lower than the percentage of CD161^+^ T cells within the CD8^+^ T-cell population.

The article "Attrition of TCR Vα7.2+ CD161++ MAIT Cells in HIV-Tuberculosis Co-Infection Is Associated with Elevated Levels of PD-1 Expression" was published in 2015. Journal: PLoS One.

**Fig 2:** Percentage of CD8^+^ T cells expressing CD161^++^ across different study groups. **(A)** Scatter plots (gated on the CD3^+^ T-cell population) show co-staining with CD8 and CD161 on representative samples from 5 different clinical groups: CPTNs, CPTPs, HVTNs, HVTPs, and HCs. **(B)** CD161^++^CD8^+^ T (MAIT cell) frequency in HCs showed significantly increased MAIT cell levels compared to other study groups. **(C)** CD161^+^CD8^+^ T cell frequency showed no difference across the different study groups. **(D-E)** CD161^++^CD8^+^ MAIT cell frequency in subjects with HIV mono-infection and HIV/TB co-infection shows no significant correlation with either HIV plasma viral load (copies/mL) or CD4^+^ T-cell counts (cells/mm^3^). All graphs show median (red bars) and range (blue whiskers); *P* values are reported for two-sided Mann-Whitney tests with threshold for significance *P* = 0.025 after Bonferroni correction for 2 comparisons. Correlations between MAIT cell frequency and markers of HIV disease progression were assessed using two-tailed non-parametric Spearman’s rank. (Note: TN, treatment naïve; TP, treatment positive; HC, healthy control; CP, HIV/TB co-infection; HV, HIV mono-infection).

### CD161^++^ MAIT Cell Frequencies do not Recover During ART and ART/ATT Therapy

Next, we sought to investigate the impact of ART and/or ATT on MAIT cells. We observed significantly reduced PVL (*P*<0.0001) and significantly increased CD4^+^ T-cell counts (*P* = 0.0004) (Table 1). However, ART-mediated viral suppression did not restore the frequency of CD161^++^ MAIT cells in HIV mono-infected treated patients (median, 1.38%; range, 0.16–3.4, *P* = 0.7) relative to HIV mono-infected treatment naïve patients (median, 0.82%; range, 0.15–6.8) and HIV/TB co-infected treated patients (median, 1.44%; range, 0.05–8.7; *P* = 0.5) in comparison with HIV/TB co-infected treatment naïve patients (median, 0.75%, range, 0.085–2.3) (Fig 2B). In addition, the HIV/TB co-infection significantly decreased the frequencies (median, 0.75%, range, 0.08–2.3) of CD161^++^MAIT cells as compared to HIV mono-infection (median, 0.82%; range, 0.15–6.8) among the treatment naïve group (Fig 2B).

### PD-1 Expressing CD161^++^ MAIT Cells Represent an Important Cellular Phenotype in HIV Mono- and HIV/TB Co-Infections

We further investigated the expression levels of PD-1 inhibitory receptor on the CD161^++^/MAIT cell populations in HIV mono- and HIV/TB co-infected patients. Our result showed that PD-1 expression was significantly increased on CD161^++^ MAIT cells of treatment naïve HIV/TB co-infected patients (median, 12.1%; range 0–33.3; *P*<0.001), treatment naïve HIV-infected patients (median, 3.2%; range, 0–27.8; *P*<0.05), and HIV-infected patients under treatment (median, 3.5%; range 0–12.8; *P*<0.05) as compared to HCs (median, 1.14%; range, 0–3.85) (Fig 3A and 3B).

The article "Attrition of TCR Vα7.2+ CD161++ MAIT Cells in HIV-Tuberculosis Co-Infection Is Associated with Elevated Levels of PD-1 Expression" was published in 2015. Journal: PLoS One.

**Fig 3:** Expression levels of different markers by CD161^++^CD8^+^ T-cell subsets in the study population. **(A)** Zebra plots of double-gating strategy (gated on the CD161^++^ CD8^+^ T cells) show staining with 4 different markers (CD103, PD-1, CCR6, CCR5) on representative samples from a HC and a CPTN. HCs showed increased amount of CCR6-expressing MAIT cells and decreased amount of PD-1 expressing MAIT cells compared to CPTNs. **(B)** HC showed significantly lower expression level of inhibitory receptor, PD-1 while HIV/TB co-infected patients show significantly increased PD-1 expressing MAIT cells. **(C)** Significantly increased CCR6-expressing MAIT cells were found in HCs compared to HIV and TB infected groups. **(D)** No significant difference was observed in CCR5 expression levels by MAIT cells among the different study subjects. The significant difference in CCR5 expression between HVTPs and HCs may be due to the limited number of samples. All graphs show median (red bars) and range (blue whiskers); *P* values are reported for two-sided Mann-Whitney tests with threshold for significance *P* = 0.025 after Bonferroni correction for 2 comparisons. (Note: TN, treatment naïve; TP, treatment positive; HC, healthy control; CP, HIV/TB co-infection; HV, HIV mono-infection).

### MAIT Cells Express Significantly Lower Levels of CCR6 During HIV/TB Co-Infection

To determine the homing capacity of CD161^++^CD8^+^ T cells, we investigated expression of homing receptors CCR6, CCR5 and the mucosal integrin receptor CD103. Majority of the MAIT cells in healthy subjects expressed a significantly higher level of CCR6 (median, 89.7%; range, 68.1–98.7) as compared to HIV/TB co-infections without treatment (median, 46.6%; range, 1.3–68.8; *P*<0.0001), HIV without treatment (median, 73.8%; range, 37.6–97.1; *P*<0.05), HIV with treatment (median, 59.7%; range, 23.4–95.6; *P*<0.001) (Fig 3C). There was no difference in the expressions of CCR5 (Fig 3D) and the integrin CD103 (data not shown).

### Attrition of TCR Vα7.2^+^CD8^+^ MAIT Cells Co-Expressing CD161 Occurs Among HIV-Infected Patients

We observed that a majority of Vα7.2 expressing cells belonged to CD161^++^ MAIT cell subset and only very negligible Vα7.2 expression was found in non-MAIT CD161^+^ (dim) and CD161^-^ T-cell subsets (Fig 1B). The frequency of Vα7.2^+^CD8^+^ T cells (MAIT cells) was significantly lower in HIV/TB co-infected patients under treatment (median, 5.6%; range, 0.28–16.7; *P* = 0.05) and HIV/TB co-infected naive treatment patients (median, 6.8%; range, 0.56–13.9; *P* = 0.05) when compared to HCs (median, 11.1%; range, 6.8–15.3) (data is not shown). However, there was no significant difference in the frequency of Vα7.2^+^CD8^+^ T cells in HIV-infected patients under treatment (median, 10.4%; range, 2.4–28.9; *P* = 0.8) and HIV-infected treatment naïve patients (median, 9.8%; range, 1.55–38; *P* = 0.3) when compared to HCs (data not shown). Interestingly, we also observed a significant decrease of CD8^+^Vα7.2^+^ MAIT cells co-expressing CD161 among HIV-infected treatment naïve patients (median, 15.7%; range, 4.2–65.2; *P* = 0.05), HIV/TB co-infected treatment naïve patients (median, 17,8%; range, 0.7–41.8; *P* = 0.001) and HIV/TB co-infected patients under treatment (median, 20.6%; range, 1.6–63.7; *P* = 0.05) as compared to HCs (median, 49.0%; range, 5.3–71.9) (Fig 4A and 4B). Conversely, a significantly higher number of CD161-CD8^+^Vα7.2^+^ MAIT cells was observed in HIV mono-infected treatment naïve patients (median, 84.1%; range, 34.5–95.7; *P* = 0.05), HIV/TB co-infected treatment naïve patients (median, 82.2%; range, 58.2–99.3; *P* = 0.001) and HIV/TB co-infected subjects under treatment (median, 79.4%; range, 36.3–97.9; *P* = 0.05) when compared to HCs (median, 50.6%; range, 28.1–93.3) (Fig 4C).

The article "Attrition of TCR Vα7.2+ CD161++ MAIT Cells in HIV-Tuberculosis Co-Infection Is Associated with Elevated Levels of PD-1 Expression" was published in 2015. Journal: PLoS One.

**Fig 4:** Profile of expression of CD161 on MAIT cells. **(A)** The zebra plots depict the gating strategy for the analysis of expression of CD161 on MAIT cells. CD8^+^ T cells were gated for TCR Vα7.2 specific for MAIT cells. After gating on CD8^+^ TCR Vα7.2^+^ MAIT cell population, CD161 expression was subsequently analyzed. **(B-C)** MAIT cells of HCs showed significant increase of CD161 compared to other infected groups. Conversely, HCs has the lowest amount of CD161^-^ MAIT cells. All graphs show median (red bars) and range (blue whiskers); *P* values are reported for two-sided Mann-Whitney tests with threshold for significance *P* = 0.025 after Bonferroni correction for 2 comparisons. (Note: TN, treatment naïve; TP, treatment positive; HC, healthy control; CP, HIV/TB co-infection; HV, HIV mono-infection).

### Surface Expression of PD-1 on CD161^++^/MAIT Cells is Inversely Proportional to the Turn-Over Rates of MAIT Cells in the Periphery

Next, we investigated if the expression of PD-1 on CD161^++^/MAIT cells had any association with the frequency of these cells in the peripheral circulation of all the study groups. Our results showed that turn-over rates of MAIT cells correlated inversely with surface PD-1 expression on CD161^++^/MAIT cells (*P* = 0.0039 and r = -0.4006) (Fig 5). This shows that PD-1 expression levels on MAIT cells likely impacts the frequency of these cells in the peripheral blood. To conclude, we hypothesized that the frequency of CD161^++^/MAIT cells correlated negatively with surface PD-1 expression on these cells.

The article "Attrition of TCR Vα7.2+ CD161++ MAIT Cells in HIV-Tuberculosis Co-Infection Is Associated with Elevated Levels of PD-1 Expression" was published in 2015. Journal: PLoS One.

**Fig 5:** Correlation analysis between PD-1 expression and CD161^++^/MAIT cell frequency in the study participants. The MAIT cells frequency correlated inversely with PD-1 expression on MAIT cells (*P* = 0.0039 and r = -0.4006). Correlation analysis between CD161^++^/MAIT cell frequencies and PD-1 expression was performed using the Spearman's rank correlation coefficient.

## Discussion

In this study, we investigated CD161^++^ MAIT cells in the peripheral blood of HIV mono- and HIV/TB co-infected subjects. We found that the number of MAIT cells was severely depleted in both HIV mono- and HIV/TB co-infected patients whereas the number of CD161^+^CD8^+^ T cells was stably maintained in patients. Our findings are in line with recent investigations [25, 27]. It has been suggested that depletion of MAIT cells could result from redistribution to other inflamed tissue sites, poor ability or failure to regenerate from thymic precursor cells, lack of antigen-presenting cells (APCs), or MAIT cell death caused by MR1-dependent antigen-induced cell death (AICD), activation-induced apoptosis, bystander cell death and direct viral infection [28].

Evidence suggests that CD161^++^ MAIT cell numbers fail to recover in the peripheral blood [26]] in spite of treatment with ARV and anti-TB drugs [28]. Our current investigation is in agreement with Leeansyah et al. in regards to the frequency of recovery of MAIT cells [26]. The effect the initiation of ART at an earlier stage of HIV infection has on MAIT cells frequency largely remains unknown and the progression rate of HIV infection damaging MAIT cell populations still remain unclear [26]. Leeansyah et al. have recently reported that the number of MAIT cells decline following exposure to HIV [26]. Here, we observed that conventional therapy increased CD4^+^ T-cell counts and decreased PVL as also reported by other investigators [25, 26] and we also found that CD161^++^ MAIT cell frequencies in subjects with HIV mono- and HIV/TB co-infections showed no significant correlation with either HIV PVL or CD4^+^ T-cell counts.

MAIT cells respond to various microbial pathogens recognized via their non-specific germline-derived TCR activated by microbial antigens [29] conferring protection from OIs. Unsurprisingly, a decline in MAIT cell frequency could impose threats to the host’s ability to deflect infection by mycobacterial, and other bacterial or fungal pathogens. This could partly explain why HIV-infected patients with lower number of MAIT cells become more prone to MTB infection although low CD4^+^ T-cells counts markedly contribute to this defect. Further, MTB can dampen MAIT cell frequency in HIV-infected patients by diverse mechanisms including accumulation in tissues and AICD [28]. This was clearly evident from our results wherein the HIV/TB co-infected group had an even lesser number of MAIT cells than the HIV mono-infected group, although our data in this aspect was not significant. Our current observation is in line with recent studies, which suggest that MAIT cell numbers in the peripheral blood of MTB-infected patients are lower as compared to normal healthy individuals and non-MTB-infected patients due to potential migration of MAIT cells to pulmonary sites to control and contain the dissemination of bacteria [7, 25]. This is also evident from the increased expression levels of MR1 on lung epithelial cells following infection with MTB [15]. Besides, there is also a possibility that HIV and MTB can contribute equally in a concerted way to decrease MAIT cell levels facilitating the chances of acquiring another infection.

The article "Attrition of TCR Vα7.2+ CD161++ MAIT Cells in HIV-Tuberculosis Co-Infection Is Associated with Elevated Levels of PD-1 Expression" was published in 2015. Journal: PLoS One.

Wong and others have also reported decreased MAIT cell numbers in HIV-negative individuals with active TB or latent TB [25]. Although MAIT cells appear to have a lesser role against viral pathogens, the role of mucosal immunity appears to be highly significant in HIV infection [30] owing to the systemic impact mucosa derived microbe-derived components has on the infection. It is clear from several studies, especially by Leeansyah that years of effective combined ART (cART) might seldom restore MAIT cell numbers in peripheral blood [19, 25, 26, 28]. Furthermore, despite the failure in numerical recovery, Leeansyah et al. have observed partial functional recovery in residual MAIT cells among HIV-infected patients following initiation of effective long-term ART [25, 26]. Exhaustion of MAIT cells in HIV-positive individuals can also be facilitated by persistent exposure to microbial antigens. MAIT cells recruitment is thought as a compensatory mechanism to defend overall CD4^+^ T-cell-depleted HIV-infected mucosa. This has been supported by the observation where MAIT cells in the rectal mucosa were better preserved than those in the peripheral blood of HIV-infected patients [26, 28].

Here, we also demonstrated that the decrease in MAIT cells frequencies might be linked to expression of PD-1 on MAIT cells. PD-1 is known for its ability to down-regulate the functional secretory abilities and proliferation of classical CD4^+^ and CD8^+^ T cells causing them to undergo functional exhaustion during persistent HIV infection [31, 32]. Nonetheless, its expression on MAIT cells has not been investigated in detail. Here, we showed that MAIT cells from healthy HCs expressed very low levels of PD-1 but the expression was significantly enhanced in HIV-infected and HIV/TB co-infected patients. Based on our finding, we propose that the decrease of MAIT cells population in HIV-mono- and HIV/TB co-infected patients is likely associated with increased expression of PD-1, which potentially induces the inhibition of MAIT cell proliferation directly or indirectly, which however remains to be investigated. Leeansyah et al. have demonstrated an increase in the levels of TIM-3 and CD57 on MAIT cells of HIV positive patients [26]. Jiang et al. have reported that MAIT cells stimulated with bacille calmette-guérin (BCG) TB antigens showed increased production of IFN-γ and TNF-α compared with HCs. However, MAIT cells stimulated with *Escherichia coli* showed lesser production of IFN-γ and TNF-α in active MTB infection. Recent research also suggests that MAIT cells in patients with active TB showed elevated expression of PD-1, and that blockade of PD-1 signaling augmented the secretion of IFN-γ in BCG-activated MAIT cells [33]. There was a negative correlation between PD-1 and MAIT cells levels in all study participants. Therefore, our results suggest that appearance of PD-1 might be linked to the decreased frequencies of MAIT cells. Interestingly, we also found that the expression of PD-1 on MAIT cells was not decreased in HIV-infected patients in spite of the initiation of treatment. However, further longitudinal studies may be required to investigate the effect of ART/ATT drugs on PD-1 expression in MAIT cells of HIV-infected patients. Of note, we also observed that both HIV mono-infected patients and HIV/TB co-infected patients had significantly increased levels of CD161^-^Vα7.2^+^CD8^+^ MAIT cells compared to HCs. Conversely, they had significantly reduced levels of CD161^+^Vα7.2^+^CD8^+^ MAIT cells in their peripheral blood when compared to healthy subjects. Similar findings have also been demonstrated by Leeansyah et al. in their recently conducted investigation [26]. This hints to the effect for the down-regulation of CD161 on MAIT cells of infected patients. Of note, increased expression of CD161 has also been correlated with the ability of MAIT cells to migrate preferentially to the intestine and liver [9]. Thus, the decline in CD161 expression implies functional defect and tissue-homing ability of MAIT cells in HIV infection.

The article "Attrition of TCR Vα7.2+ CD161++ MAIT Cells in HIV-Tuberculosis Co-Infection Is Associated with Elevated Levels of PD-1 Expression" was published in 2015. Journal: PLoS One.

CCR6 is a chemokine receptor that may play a role in trapping CCR6^+^ T cells in secondary lymphoid tissues due to increased CCR6 ligand production during HIV infection [26]. It has been suggested that the trapped cells then undergo apoptosis leading to the gradual loss of CCR6^+^ T cells. Thus, CCR6 can be used as a marker to monitor HIV disease progression [34]. CCR6 is also one of the characteristics for a specific population of memory cells that secrete TNF-α, IL-2, and IFN-γ upon infection [34]. In our study, the significant decrease of CCR6 expression on MAIT cells of HIV mono-infected and HIV/TB co-infected patients may explain why HIV-infected patients have weakened immunity at their mucosal sites, especially at genitalia, respiratory, and intestinal mucosal surfaces. CCR5 is a chemokine receptor that has been well described as a HIV entry co-receptor on CD4^+^ T cells [35]. We didn’t observe so much difference in the number of MAIT cells expressing CCR5 among the different study groups. This is in contrast to another recent study, which demonstrated the high level expression of CCR5 by MAIT cells of healthy individuals [25]. They also showed significantly lesser expressions of CD103 on MAIT cells in HCs, which on the other hand was not significant in our current investigation.

In conclusion, our study showed that MAIT cells frequency was severely depleted during HIV mono- and HIV/TB co-infections. This observation is important as it suggests that MAIT cells may have significant roles in HIV infection besides bacterial and fungal infections. Further investigations with tissue samples of HIV-infected patients may be necessary to deduce the precise role of recruitment of MAIT cells in HIV infection. Moreover, PD-1 was highly expressed on MAIT cells in the peripheral blood of HIV mono- and HIV/TB co-infected patients, and that this elevated expression was not decreased in spite of initiating treatment with ART/ATT drugs, suggesting that these cells undergo immune exhaustion as a consequence of HIV infection. Our data supports a role for a functional role of MAIT cells in innate defense against HIV infection, and is vulnerable to immune exhaustion as a consequence of HIV infection. Decrease of CCR6 expression likely explains why HIV-infected patients have weakened mucosal barrier immunity attributes.
